# Anatomical and Biochemical Traits Related to Blue Leaf Coloration of *Selaginella uncinata*

**DOI:** 10.1155/2022/1005449

**Published:** 2022-02-24

**Authors:** Lin Li, Lulu Yang, Aihua Qin, Fangyi Jiang, Limei Chen, Rongyan Deng

**Affiliations:** ^1^College of Architectural Arts, Guangxi Arts University, Nanning 530007, China; ^2^Forestry College, Guangxi University, Nanning 530004, China

## Abstract

*Selaginella uncinata* shows particularly rare blue leaves. Previous research has shown that structural interference by the cell wall of adaxial epidermal cells imparts blue coloration in leaves of *S. uncinata*; the objective of this study was to see whether anthocyanins might additionally contribute to this color, as changes in pH, and conjugation with metals and other flavonoids is also known to result in blue coloration in plants. We compared anatomical and biochemical traits of shade-grown (blue) *S. uncinata* leaves to high light (red) leaves of the same species and also to a non-blue (green) leaves of a congeneric *S. kraussiana*. By examining the anatomical structure, we found that the shape of adaxial epidermis of *S*. *uncinata* leaves was convex or lens-shaped on the lateral view and irregular circles with smooth embossment on the top view. These features were different from those of the abaxial and adaxial epidermis of *S*. *kraussiana*. We suspect that these structures increase the proportion of incident light entering the cell, deepening the leaf color, and therefore may be related to blue leaf color in *S*. *uncinata*. By examining biochemical traits, we found little difference in leaf pH value among the leaf types; all leaves contained several metal ions such as Mg, Fe, Mn, and copigments such as flavones. However, because there was no anthocyanin in blue *S*. *uncinata* leaves, we concluded that blue coloration in *S. uncinata* leaves is not caused by the three hypotheses of blue coloration: alkalization of the vacuole pH, metal chelation, or copigmentation with anthocyanins, but it may be related to the shape of the leaf adaxial epidermis.

## 1. Introduction

Colorful leaves are attractive features that characterize ornamental plants. Red, purple, yellow, and variegated leaves are common, whereas blue leaves are particularly rare. *Selaginella uncinata*, a fern species that is adapted to the shaded conditions, is such a blue leaf plant. It has a blue upper and green lower surface. There have been some reports related to *S. uncinata* focusing on structural anatomy [1], developmental anatomy [2], cell genetics [3], chloroplast genome [4–6], and chemicals and medicine [7–13]. Our previous research showed that the leaf color of *S. uncinata* appears normally blue in the shade, while it changes to red under full light exposure [14], and this color change under high light corresponded with a reduction in chlorophyll and anthocyanin and an increase in carotenoids, resulting in a dominant orange color. Based on the transcriptome sequencing and quantitative real-time polymerase chain reaction (qRT-PCR) analysis, we concluded that the primary pathway of pigment metabolism in *S. uncinata* may be the chlorophyll metabolism pathway rather than the anthocyanin biosynthesis pathway [15]. According to the research of leaf coloration mechanism, leaf coloration in plants can be due to either pigments or structural coloration. These two groups differ in their appearance—pigmented colors look the same from all angles, while structural colors appear with different hues when viewed from different angles, a unique attribute of structural color called iridescence [16].

There have been very few studies on the production of blue leaves. Hébant and Lee [1] found that the iridescent blue color of *S. uncinata* and *S. willdenowii* is caused by thin-film interference (a physical effect). In other blue iridescent plants, the iridescent ultrastructural basis is relevant to their adaxial epidermis, but they are different in detail. In *Diplazium tomentosum*, *Lindsaea lucida*, and *Danaea nodosa*, the iridescent ultrastructure is that in the uppermost cell walls of the adaxial epidermis, the arrangement of multiple layers of cellulose microfibrils is helicoidal [17, 18]. In *Begonia pavonina*, *Phyllagathis rotundifolia*, and *Elaeocarpus angustifolius*, blue coloration is due to the parallel lamellae in specialized plastids (iridoplasts) adjacent to the abaxial wall of the adaxial epidermis [18, 19], while in *Trichomanes elegans,* it results from the remarkably uniform thickness and arrangement of grana in specialized chloroplasts adjacent to the adaxial wall of the adaxial epidermis [17]. In these studies, it was not possible to extract blue pigment from the study material, such that in all cases, blue iridescence was considered to be a structural color.

However, according to studies of blue flowers, pH in the vacuole [20–22], metal chelation [23], and copigmentation [24, 25] may also be related to blue coloration. It seems clear that blue leaves in *S*. *uncinata* have a structural mechanism, but whether it is also affected by any or all of these three factors remains unknown. In our previous study, we detected low content of anthocyanins in *S. uncinata* [14]. The objective of this study was to further investigate the possibility that anthocyanins may contribute to blue coloration in *S. uncinata*, by examining leaf pH, metal ions, and pigment composition, in addition to anatomical structure.

## 2. Material and Methods

### 2.1. Plant Material

We conducted tests on three leaf types: blue *S. uncinata* leaves grown under a sunshade net (light intensity: 65–105 umol m^−2^ s^−1^), green S. kraussiana leaves grown under the same conditions, and red S. uncinata leaves grown in full exposure (light intensity: 500–520 umol m^−2^ s^−1^) [14]. There were 6 POTS for each leaf type and 3 replicates for a total of 54 POTS. All plants were 6 months old, given normal water and fertilizer management, and cultivated in the nursery of the Forestry College, Guangxi University, Nanning, China. Mature normal leaves were selected randomly in different directions from various individuals when sampling.

### 2.2. Methods

We compared observations within species (blue and red *S. uncinata* leaves) and between species (blue *S. uncinata* and green *S. kraussiana* leaves). The traits examined included morphology, color parameters, leaf paraffin transverse sections, freehand sections, and scanning electron microscopy (SEM) photomicrographs to determine the structural mechanism. We also compared reported leaf pH values, and metal ion, anthocyanin, and flavonoid content to examine the physiological and biochemical mechanisms related to blue coloration.

### 2.3. Anatomical and Morphological Traits

#### 2.3.1. Morphological Traits and Leaf Color Parameters

Morphological observations and measurements included leaf type, leaf texture, leaf color on the adaxial and abaxial sides, leaf size, and leaf thickness. The procedure is repeated 6 times, and the results are averaged.

Fresh leaves are taken, and leaf color in the middle of the upper epidermis was measured by Royal Horticultural Society Colour Chart (RHSCC) and a General Colorimeter (NR10QC, 3nh, Shenzhen). In a daylight condition, lightness (*L*^*∗*^) and two chromatic components *a*^*∗*^ and *b*^*∗*^ of the CIEL^*∗*^*a*^*∗*^*b*^*∗*^ color coordinate were measured. Based on the equations: *C*^*∗*^=(*a*^*∗*2^+*b*^*∗*2^)^1/2^ and *h* = arctan (*b*^*∗*^/*a*^*∗*^), chroma (*C*^*∗*^) and hue angle (*h*) were calculated. The procedure is repeated 5 times, and the results are averaged.

#### 2.3.2. Microscopic Observation of Leaf Transverse Sections

The transverse sections of leaves were prepared according to Li [26]. Leaves were collected and fixed in a formalin-acetic acid-alcohol (FAA; absolute ethyl alcohol: glacial acetic acid, 3 : 1) solution for 30 min; fixed samples were washed three times in 50% ethanol and dehydrated through a series of ethanol concentrations: 60% (30 min), 70% (30 min), 85% (30 min), 95% (5 min), and 100% (5 min, twice). Ethanol in dehydrated samples was then replaced with xylol and paraffin, and samples were embedded and cut into sections of 8–14 *μ*m thickness using a fully motorized rotary microtome (Leica RM2245, Germany). The sections were stained with Safranin Fast Green, washed with 50% ethanol, and then observed with a digital microscope (×10) (Nikon Eclipse E100, Japan).

#### 2.3.3. Microscopic Observation of Leaf Epidermal Cells

Freehand sections were prepared for leaf shape observations. We rinsed 1.5 × 2 cm leaf samples with distilled water, put them into a 1 : 1 solution of glacial acetic acid and 30% peroxide water, and then placed them in a 60°C incubator for 2–3 h. The samples were rinsed with distilled water, and peels (at least 2 mm long) of the upper and lower surfaces were made with fine-tipped tweezers from the central area of a single leaf and mounted in water, stained with Safranin for 30–60 s, washed, and observed with a digital microscope (Nikon Eclipse E100) [27].

#### 2.3.4. Scanning Electron Microscopy

Leaf epidermal three-dimensional structure was observed by SEM (Hitachi, S-3400N, Japan). 1.5 × 2 cm samples from each of the three samples were cut, respectively, from the middle of each leaf and fixed with 2.5% glutaraldehyde solution for 2 h at room temperature, rinsed with 0.1 mol L^−1^ phosphate saline buffer, and dehydrated through increasing alcohol series, and then, the alcohol was replaced with isoamyl acetate. The samples were dried naturally, cut into appropriate sizes, and coated using a sputter coater. They were subsequently observed and photographed using SEM [28].

### 2.4. Physiological and Biochemical Traits

#### 2.4.1. Measurement of Leaf pH

The three samples were collected and rinsed, and 5 g of leaves was weighed and cut into pieces. We then added 50 ml distilled water, vibrated the samples for 10 min after soaking for 12 h, and measured the pH of the solution at 30°C using a pH meter (PHS-25, Hongyi, Shanghai) [29]. The procedure is repeated 3 times, and the results are averaged.

#### 2.4.2. Leaf Metal Ion Measurements

Dried leaves were ground into a fine powder, and a 0.6 g sample of dried material was digested in 5 ml of concentrated HNO_3_ and 1 ml of H_2_O_2_, followed by the treatment in a high-performance microwave digestion unit (CEM, Mars, Matthews, NC, USA). Settings used were as follows: time (minutes)/power (watts)/temperature (°C): 5/1,200/120, 10/1,200/160, and 20/1,200/180. After complete digestion and acid removal, the samples were diluted with ultrapure water for measurement. The procedure is repeated 3 times, and the results are averaged. Sample solutions were analyzed for elements by ICP-MS (NexION 350X, PerkinElmer, Waltham, MA, USA). The parameters for analysis were as follows: plasma power: 1,400 W, plasma flow: 18 l/min, auxiliary flow: 1.8 l/min, and sampling depth: 7.5 mm [30].

#### 2.4.3. Anthocyanin Analysis

Only blue leaf samples were analyzed for anthocyanin components using ultra-performance liquid chromatography (UPLC). The methods of extraction were as previously described [31] with some modifications. Anthocyanins were extracted from 0.5 g freeze-dried leaf powder from blue leaves in 25 ml of 2% formic acid/methyl alcohol for 24 h at 4°C. The supernatant was removed and stored under the same conditions. The extraction was repeated once. These two extractions were merged and subjected to rotary evaporation at 30°C until the anthocyanins were dry. We then added a moderate amount of 2% formic acid solution to dissolve the residue and ethyl acetate to extract the anthocyanins in the aqueous phase.

A 20 *μ*L sample was quantified by UPLC-triple-time-of-flight/mass spectrometry (TOF/MS) (Acquity^TM^ Ultra, Waters, Milford, MA, USA) at a flow rate of 0.8 ml/min and a column temperature of 30°C using a 4.6 × 100 mm column of C18 and a linear gradient of solvent A (0.1% formic acid/water (v/v)) in solvent B (acetonitrile) for 30 min. The detection was performed by absorption at 520 nm. The gradient settings were as follows: 0 min, 10% B; 5 min, 10% B; 20 min, 40% B; 25 min, 100% B; and 30 min, 10% B.

#### 2.4.4. Flavonoid Analysis

The extraction methods as previously described by Zhu et al. [27] were referenced with some modifications. Flavonoids were extracted from 1.0 g freeze-dried leaf powder from three 2% formic acid/methyl alcohol samples, after oscillation in ultrasonic cleaners for 20 min at 20°C, and clarified by centrifugation at 12,235 × *g* for 10 min. The supernatant was then collected. The extraction was repeated twice, and the total extraction volume was 25 ml. After the combined extraction was filtered with a 0.22 *μ*m nylon microporous filter, the solution was tested.

UPLC conditions are as follows: a 5 uL sample was quantified by UPLC-Triple-TOF/MS (Acquity^TM^ Ultra, Waters) at a flow rate of 0.8 ml/min and a column temperature of 30°C using a 4.6 × 100 mm column of C18 and a linear gradient of solvent A (0.1% formic acid/water (v/v)) in solvent B (0.1% formic acid/acetonitrile (v/v)) for 38 min. The detection was performed by absorption at 280 nm. The gradient settings were as follows: 0 min, 5% B; 2 min, 5% B; 25 min, 50% B; 35 min, 95% B; 37 min, 95% B; and 38 min, 5% B.

MS was performed on an UPLC-Triple-TOF 5600 Plus System (AB Sciex, Framingham, MA, USA) equipped with an electrospray ionization source (ESI) system. The optimal MS conditions were as follows: scan range m/z of 100–1500. The experiment was conducted in negative ion mode, with a source voltage of −4.5 kV and source temperature of 550°C. The pressure of both gas 1 (air) and gas 2 (air) was set to 50 psi. The pressure of curtain gas (N2) was set to 35 psi. The maximum allowed error was set to ±2 ppm. The collision energy was 40 V, with a collision energy spread of 20 V. Exact mass calibration was performed automatically before each analysis, employing the automated calibration delivery system.

## 3. Results

### 3.1. Anatomical and Morphological Traits

#### 3.1.1. Morphological Traits and Leaf Color Parameters

Blue *S. uncinata* leaves were soft and thin; newly formed leaves were grass green. The adaxial side of mature leaves was glaucous, showing iridescence (Figure 1(a)), whereas the abaxial side was green (Figure 1(b)). Red *S. uncinata* leaves were hard and crisp; newly formed leaves were also grass green, and the adaxial and abaxial sides of the mature leaf were red (Figures 1(c) and 1(d)). *S. kraussiana* leaves were thick and soft; newly formed leaves and the adaxial and abaxial sides of mature leaves were all green (Figures 1(e) and 1(f)).

The measurement data for the three samples are shown in Table 1. The results indicated that the thickness of red leaves was significantly greater than that of blue leaves, whereas the area of blue leaves was significantly greater than that of red leaves.

The color parameters for the three samples are shown in Table 2. The results indicated that their hue angles (*h*) are all near 0° and belong to the red-purple area. The chroma (*C*^*∗*^) of blue leaves was significantly greater than that of red leaves.

Note: data analysis used Duncan's method, and the data of *L*^*∗*^*a*^*∗*^*b*^*∗*^ = mean value ± standard deviation (*n* = 5); A and B show the different significant differences at *P*=0.05 level in SNK test.

#### 3.1.2. Anatomical Structure of Leaf Transverse Section

The anatomical structure was observed in leaf transverse sections by the paraffin section. The three leaf types shared some similar features: the epidermis is covered by the cuticle; between the upper epidermis and the lower epidermis are irregularly shaped mesophyll cells; and there is no obvious differentiation of palisade and spongy tissue in the mesophyll. There are large chloroplasts in the mesophyll cells; these are long, narrow, and moniliform distribution. Cell arrangement is loose, with large gaps between the cells, forming well-developed aeration tissue in the mesophyll cells.

The shapes of leaf adaxial and abaxial epidermal cells in blue and red *S. uncinata* were different from *S. kraussiana*. The shape of leaf adaxial and abaxial epidermal cells was different in blue leaves: the adaxial epidermis consisted of convex or lens-shaped cells, whereas the abaxial epidermis consisted of long cylindrical cells on the lateral view. In blue leaves, chloroplasts were distributed in the upper and lower epidermal cells, and in mesophyll cells, they were mainly at the bottom of the upper epidermal cells (Figure 2(a)). The shape of leaf adaxial and abaxial epidermal cells in red leaves was similar to that of blue leaves; however, the cells were much more closely aligned, and chloroplasts were significantly reduced (Figure 2(b)). The leaf adaxial and abaxial epidermal cells in *S*. *kraussiana* were long and cylindrical on the lateral view. Chloroplasts were distributed in the upper and lower epidermal and mesophyll cells, but primarily in the mesophyll cells (Figure 2(c)).

### 3.2. The Shape of Epidermal Cell

We used the freehand section to observe epidermal cells from the upper face and SEM photomicrographs to observe the three-dimensional shape of the epidermal cells. We found that the shapes of leaf adaxial and abaxial epidermal cells in blue *S*. *uncinata* were different: the adaxial epidermis was irregular circles, with smooth embossment, and by contrast, the abaxial epidermis was a long, wavy, irregular strip, with elongated embossment on the top view (Figure 3(e)). The shape of leaf adaxial and abaxial epidermal cells in red leaves was similar to that of blue leaves (Figure 3(f)). The leaf adaxial and abaxial epidermal cells in *S*. *kraussiana* were both shaped as irregular long strips, with elongated embossment on the top view (Figure 3(g)).

### 3.3. Physiological and Biochemical Traits

#### 3.3.1. Leaf pH

Leaf pH values were in the range of 4.5–5.0 (Table 3), in the order blue *S*. *uncinata* leaves > red *S*. *uncinata* leaves > *S*. *kraussiana* leaves. The pH value of blue *S*. *uncinata* leaves was significantly greater than that of other two.

#### 3.3.2. Leaf Metal Ion Content

Mg ions were very abundant in all three leaf types (>3000 mg/kg). The Ca, Mn, Fe, Zn, and Al ion contents were also relatively high (55–1200 mg/kg). There was little Cu ion content (<9 mg/kg). Cd ion content was the lowest, ranging from 0.03 to 0.04 mg/kg (Table 4).

#### 3.3.3. Anthocyanin Analysis

The extract solution in blue *S*. *uncinata* leaves contained no anthocyanins (Figure 4). No anthocyanin ion peaks were observed through mass spectrometry. The result is in line with our conclusion that was previously published: the primary pathway of pigment metabolism in *S*. *uncinata* might not be the anthocyanin biosynthesis pathway, but rather the chlorophyll metabolism pathway [15].

#### 3.3.4. Flavonoid Analysis

There was good flavonoid separation among the three leaf types (Figures 5–7). We compared the peaks on the chromatographic map and the results of the mass spectrogram, total ion flow diagram, and debris ion mass spectrum analysis to the SciFinder and Reaxys databases and finally inferred 15, 20, and 9 types of flavonoids in blue *S*. *uncinata* leaves, red *S*. *uncinata* leaves, and *S*. *kraussiana* leaves, respectively (Figure 8 and Table 5).

#### 3.3.5. Comparison of Flavonoid Composition in the Three Leaf Types

There are 7 common compounds in the three leaf types: apigenin 6,8-di-C-*α*-L-arabinopyranoside, amentoflavone, robustaflavone, 2,3-dihydrorobustaflavone, bilobetin, robustaflavone 4′-methyl ether, and 4′,7“-di-O-methylamentoflavone.

We find that the vast majority of the flavonoids present (14 compounds) in blue and red leaves are similar; the component specific to blue leaves was genistein, which has an antioxidant effect. Components specific to red leaves were 6,8-C-diglucosylapigenin, apigenin 6,8-di-C-*α*-L-arabinopyranoside, apigenin 6,8-di-C-*α*-L-arabinopyranoside isomeride, 3-O-methylamentoflavone, dihydrobilobetin, and dihydrorobustaflavone 4'-methyl ether. These components are likely to play an adaptive role in high light intensity *S*. *uncinata* environments.

The results show that most of the flavonoids (7 compounds) in blue *S*. *uncinata* leaves and *S*. *kraussiana* leaves are similar. The components specific to blue leaves were 6-C-arabinosyl-8-C-glucosylapigenin, genistin, genistein, 2“,3“-dihydroamentoflavone, 2,3,2“,3“-tetrahydroamentoflavone, 2,3-dihydroamentoflavone, 2,3,2“,3“-tetrahydrorobustaflavone, and 7“-O-methyl-2,3,2“,3“-tetrahydrohinokiflavone. Among these, genistin and genistein are isoflavones. The components specific to *S*. *kraussiana* were 3-O-methylamentoflavone and robustaflavone 4'-methyl ether isomeride.

#### 3.3.6. Comparison of Blue *S. uncinata* Leaf Flavonoid Composition with Published Values

Zheng et al. [9] identified seven types of flavonoids using high-performance liquid chromatography (HPLC), modern spectroscopy, and nuclear magnetic resonance (NMR). Four of these were consistent with our results: amentoflavone, 2“, 3“-dihydroamentoflavon“, 2,3,2“,3“-tetrahydroamentoflavone, and 2,3-dihydroamentoflavone. Yiet al. [32] also identified 2,3-dihydroamentoflavone. Of the five identified types of flavonoids detected by [33] through Sephadex LH-20, chromatography, UV, and MS, those in common with our findings were as follows: amentoflavone, robustaflavone, and 7“-O-methyl-2,3,2“,3“-tetrahydrohinokiflavone. However, there was no common constituent between the studies of Wuet al. [34] and this study. In conclusion, flavonoids identified in blue *S*. *uncinata* leaves were similar to those found in previous studies; others were slightly different in structure.

## 4. Discussion

### 4.1. The Adaptability of Leaf Morphology and Anatomical Structure to Environmental Conditions

Leaf thickness is an important indicator of plant shade tolerance. Thinner leaves make fern chloroplasts more fully capable of absorbing light energy; improving the photosynthetic efficiency of ferns; and making them better adapted to shaded environments [35]. Morphology traits and measurement data show that blue *S*. *uncinata* leaves, including increased leaf area and decreased leaf thickness, are adaptations to low-light environments and weak-light intensity.

Many researchers consider that shade-tolerant trees have a greater ability to change their leaf anatomical structure [36]. Leaf anatomical structure traits such as wax coating, shape of epidermal cells, epidermal thickness, and epidermal hair play an important role in light absorption, even determining the light use efficiency of the plant [37]. Deep-shade plants change their morphology and physiology traits of cells and chloroplasts to fit the low-light conditions [38]. In the paraffin sections of the three leaf types, we observed no clear differentiation of the palisade and spongy tissues in the mesophyll, and mesophyll cells were irregularly distributed. This trait contributes to reducing projection loss of quantum light, allowing the plant to fully utilize limited light to carry out photosynthesis and accumulate organic matter, thus adapting to the shaded environment [35].

Previous research has shown that fern mesophyll cells possess more intercellular space, forming well-developed aeration tissue that can be used to store gases for photosynthesis and respiration, to make up for deficiencies in gas absorption, which is also an adaptation to a shaded environment [35]. The chloroplast is the main site of photosynthesis; in ferns, this structure appears long and narrow and is distributed as a moniliform, reducing the amount of photons penetrating the leaf and raising the utilization rate of quantum light in weak-light conditions, to improve the efficiency of leaf photosynthesis [35]. Plant chloroplasts typically exist in mesophyll cells, but through paraffin section observation, we found that chloroplasts in blue *S*. *uncinata* leaves exist mainly in epidermal cells and are larger. This result is consistent with that of Hébant and Lee [1], who examined transverse leaf sections of *S*. *uncinata* by light microscopy, but is different from those of Sheue et al., and they found several chloroplasts in the mesophyll cells and the ventral epidermal cells, while only one single giant chloroplast (bizonoplast, BP) per dorsal epidermal cell [39]. The preferential localization of chloroplasts in the lower part of the epidermal cells in *S*. *uncinata* would allow more light to penetrate and reach mesophyll cells [39], which is an adaptation of plants to weak-light environments.

### 4.2. Effects of the Shape of Leaf Epidermal Cells on Blue Coloration in *S. uncinata*

The shape of petal epidermal cells has a great influence on the formation of flower color. Noda et al. [40] found that a conical shape in the epidermal cells of petal was believed to enhance light absorption and thus intensified its color, while the flat shape could reflect more incident light and thus lightened its color. Quintana et al. [41] found that in *Anagallis*, the epidermis contains anthocyanins, and most epidermal cells are flat, with dome-shaped and conical cells in the outer layer. Mudalige et al. inspected the perianths of 34 *Dendrobium* Sw. species and hybrids to clarify the relevance of pigment distribution, the shape of upper epidermal cells, color intensity, perception, and visual texture [42]. Four types of epidermal cell shapes were identified in these *Dendrobium* flowers: flat, dome-shaped, elongated dome-shaped, and papillate [42]. Yue [43] observed using SEM measurements that the epidermal cell shapes of 17 monocotyledon flowers could be grouped into five classes: conical, flat, oval, strip-shaped, and irregular mosaic. That study suggested that convex epidermal cells increased the refraction of light, making petal color appear deeper, and that bulging cells appeared to be more conducive to pigment, whereas flat epidermal cells decreased the effect, making their color appear lighter.

By comparing leaf paraffin transverse sections, freehand sections, and SEM photomicrographs, we found that the shape of the adaxial epidermis of *S*. *uncinata* leaves was not only different from the abaxial epidermis, but also different from the adaxial epidermis of *S*. *kraussiana*. The shape appeared convex or lens-shaped on the lateral view and irregular circles with smooth embossment on the top view. This result corresponds with those of Hébant and Lee [1], who examined the convexly curved upper epidermal cells of *S*. *willdenowii* by SEM. The structure increases the proportion of incident light entering the cell, deepens the leaf color [40, 43], and therefore may be related to blue leaf coloration.

According to Hébant and Lee [1], the blue color of *S. uncinata* results from thin-film interference. Which contributes more to blue coloration? Is it thin-film interference or convex or lens-shaped epidermal cells? Do they work complementary? It needs more intensive research.

### 4.3. Effects of the pH on Blue Coloration in *S. uncinata*

The color of plant leaves is affected to some extent by the pH within vacuoles, which has a great influence on the coloration of anthocyanins, with varying performance among different plant species. Tang et al. [44] found that the pH affected anthocyanin synthesis and stability. The degradation rate of anthocyanins has been accelerated by increasing the pH during the process of red turning green in *Loropetalum chinense* var. *rubrum*. Studies on the relationship between leaf pigment content and leaf color change in *Liquidambar formosana* have shown that a reduction in pH was one reason their leaves turned red [45]. Research by Shi [46] indicated that *Prunus cerasifera* leaf color appeared red in a medium with pH <5, and the stronger the acidity, the more red the pigment. Red color was stable when the pH ranged from 4 to 5, and the solution turned green at pH >5. The stronger the alkalinity, the more green the pigment. Most research results have indicated that anthocyanins present stable red when the pH of the vacuole is lower, and unstable blue occurs as the pH increases.

The vacuole is the largest organelle in the mature leaf cell. The pH of leaf juice is often used to approximate the pH of the vacuole [47]. We used this method in our experiment, with results indicating that the pH of blue leaves was greater than that of red leaves. This result is consistent with previous results that the pH of blue flowers was greater than that of red flowers, in *Hydrangea macrophylla* [48] and *Pharbitis nil* (Linn.) *Choisy* [22]. However, for the specific value, the difference between the two pH values was only 0.08, and the difference between those of blue *S*. *uncinata* leaves and *S*. *kraussiana* leaves is only 0.11, whereas that between blue and red cultivars of *H*. *macrophylla* was 0.8 [48] and that between blue in the full-bloom stage and red in the burgeoning stage of *P*. *nil* (Linn.) *Choisy* was 1.1 [22]. Therefore, we conclude that blue leaf coloration in *S*. *uncinata* has no concern with alkalization of the pH in the vacuole.

### 4.4. Effects of Metal Ion Content on Blue Coloration in *S. uncinata*

#### 4.4.1. Effects of Metal Ion Content on Anthocyanin Coloration

Anthocyanins can be combined with metal ions and flavonoids in a stoichiometric ratio or not, to be assembled into metal pigment complexes [49], and these complexes can affect the coloration of plant leaves. There have been several studies of metal anthocyanins making color tend toward bluish, and these concentrate primarily on Mg, Al, Fe [23–25, 48, 50], Ca [30], and Mn [30]. Metal ions have a stable and protective effect on anthocyanins, and the pigments are often chelated if the cell sap contains metal ions such as Al, Fe, Mg, or Mo. In particular, anthocyanins, which change their color to some degree, often tend toward purple after chelation [51].

In our experiment, Mg, Ca, Mn, Fe, Zn, and Al ion contents were all relatively high in the three leaf types; however, there was no anthocyanin in blue *S*. *uncinata* leaves, so we concluded that blue leaf coloration in *S*. *uncinata* was unrelated to metal chelation with anthocyanin.

#### 4.4.2. Effects of Metal Ion Content on Chlorophyll

Metal ions insert protoporphyrin IX, which is the branching point of chlorophyll synthesis and heme and plant pigment synthesis, Mg ions under the catalysis of a Mg ion chelating enzyme (CHLH) insert protoporphyrin IX, forming the chlorophyll branch; Fe ions under the catalysis of a Fe ion chelating enzyme (FECH) insert protoporphyrin IX, forming the heme and plant pigment branch. At the branch point, CHLH and FECH complete protoporphyrin IX [52].

Mg is a part of the molecular composition of chlorophyll; chlorophyll formation will be affected if it is lacking. The concentration of Mg^2+^ influences the activity of CHLH [53]. Fe is necessary for protochlorophyllide formation; Mg-protoporphyrin IX and Mg-protoporphyrin IX methyl ester accumulate when short of Fe, and protochlorophyllide cannot form chlorophyll [53, 54]. Chlorophyll synthesis is also affected by the content of Cu, Mn, and other ions.

In our experiment, the Cu content was not high, but those of Mg, Fe, and Mn were very high, particularly that of Mg, with content reaching 4311.7 mg/kg, which was 1.24-fold higher in blue leaves than in red leaves. We speculate that such high Mg levels may be associated with chlorophyll synthesis in *S*. *uncinata.*

### 4.5. Effects of Anthocyanin and Copigment on Blue Coloration in *S. uncinata*

Copigments, often flavone and flavonols, are the two branches of the flavonoid metabolic pathway [55]. Combined with anthocyanins, they can stabilize pigments, and the compounds they form will influence the coloration of anthocyanins to some degree [56]. Research by Li [57] found that the effect of copigments turned purple or pink delphinidin flowers blue. Malvidin-3-glucoside is the basic anthocyanin of *Primula sinensis*; the flower appears purple when it is combined with flavonol, but appears garnet when not combined [58]. Under certain conditions, the larger the molar ratio of flavonols and anthocyanins, the more significant the copigmentation effect.

In our research, we detected anthocyanins in a preliminary experiment by measuring absorbance values using an enzyme-linked immunosorbent assay (ELISA). Although the overall content was low, and the highest content was only 1.2 pigment units [14], we still initially speculate that blue leaf coloration in *S*. *uncinata* may be related to delphinidin in anthocyanins, or a copigment with anthocyanins. We did not detect anthocyanins in blue leaves using liquid chromatography-MS (this is accordant with the conclusion that compared with the anthocyanin biosynthesis pathway, the chlorophyll metabolism pathway may be the primary pigment metabolism pathway of *S. uncinata* [15], although there were copigments such as flavone). If anthocyanins are not present, the copigmentation of flavone cannot occur. Therefore, we infer that blue leaf coloration in *S*. *uncinata* was not caused by copigmentation of anthocyanins.

## 5. Conclusion

Through comparison of leaf paraffin transverse sections, freehand sections, and SEM photomicrographs, we found that the shape of the adaxial epidermis of *S*. *uncinata* leaves was convex or lens-shaped on the lateral view and irregular circles with smooth embossment on the top view. These shapes were different from those on the abaxial epidermis and the adaxial epidermis of *S*. *kraussiana* leaves. We speculated these structures increase the proportion of incident light entering the cell, deepening the leaf color, and therefore may be related to blue leaf coloration.

Through comparison of previously published values of leaf pH and metal ion content, anthocyanins, and flavonoids with those of the three leaf types in our study, we found that leaf pH was similar among the leaf types and that the leaves all contained high levels of metal ions such as Mg, Fe, Mn, and copigments such as flavones. However, because there was no anthocyanin present in blue *S*. *uncinata* leaves, we conclude that blue leaf coloration in *S*. *uncinata* was not related to the three hypotheses of blue coloration: alkalization of vacuole pH, metal chelation, and copigmentation with anthocyanins.

## Figures and Tables

**Figure 1:** Appearance of the three leaf types. (a) Adaxial sides of blue *Selaginella uncinata* leaves; (b) abaxial sides of blue *S. uncinata* leaves; (c) adaxial sides of red *S. uncinata* leaves; (d) abaxial sides of red *S. uncinata* leaves; (e) adaxial sides of *S. kraussiana* leaves; and (f) abaxial sides of *S. kraussiana*.

**Figure 2:** Leaf paraffin transverse sections of the three leaf types. (a) Blue *S. uncinata* leaf; (b) red *S. uncinata* leaf; and (c) *S*. *kraussiana*.

**Figure 3:** Leaf epidermal cell shape of the three leaf types. (a) Freehand section photomicrographs of adaxial epidermis; (b) freehand section photomicrographs of abaxial epidermis; (c) SEM photomicrographs of adaxial epidermis; (d) SEM photomicrographs of abaxial epidermis; (e) blue *S*. *uncinata* leaf; (f) red *S*. *uncinata* leaf; and (g) *S*. *kraussiana*.

**Figure 4:** Chromatogram (520 nm) and total ion flow diagrams for anthocyanin extracting solution in blue *S*. *uncinata* leaves. Note: the peaks near 28 min are solvent background peaks.

**Figure 5:** Ultraviolet (280 nm) chromatogram and total ion flow diagrams of flavonoid extracting solution for blue *S. uncinata* leaves.

**Figure 6:** Ultraviolet (280 nm) chromatogram and total ion flow diagrams of flavonoid extracting solution for red *S. uncinata* leaves.

**Figure 7:** Ultraviolet (280 nm) chromatogram and total ion flow diagrams of flavonoid extracting solution for *S. kraussiana* leaves.

**Figure 8:** Venn diagram of flavonoids in the three leaf types.

**Table 1:** Morphological comparison of the three leaf types.

Leaf type	Leaf texture	Leaf thickness (*μ*m)	Leaf area		
			Length (mm)	Width (mm)	LW^−1^
Blue *S*. *uncinata* leaves	Soft and thin	48.53 ± 3.56B	3.25 ± 0.61C	1.73 ± 0.44C	1.9
Red *S*. *uncinata* leaves	Hard and crisp	84.34 ± 4.62C	3.09 ± 0.63A	1.53 ± 0.27B	2.0
*S*. *kraussiana* leaves	Thick and soft	35.73 ± 3.05A	3.20 ± 0.32B	1.37 ± 0.34A	2.4

Note: data analysis used Duncan's method, the data of leaf thickness, and length and width = mean value ± standard deviation (*n* = 6); A, B, and C show the different significant differences at *P*=0.05 level in SNK test.

**Table 2:** Color parameters of the three leaf types.

Leaf type	RHSCC (A)	*L* ^*∗*^	*a* ^*∗*^	*b* ^*∗*^	*C* ^*∗*^	h/°
Blue *S*. *uncinata* leaves	120	88.87 ± 0.83B	−0.85 ± 0.21A	−1.31 ± 0.10A	1.57 ± 0.19B	1.01 ± 0.09A
Red *S*. *uncinata* leaves	59	81.35 ± 6.34A	0.00 ± 0.35B	−0.46 ± 0.73B	0.83 ± 0.26A	0.69 ± 1.27A
*S*. *kraussiana* leaves	141	85.61 ± 3.90AB	−0.42 ± 0.48AB	−0.97 ± 0.39AB	1.09 ± 0.53AB	0.66 ± 1.23A

**Table 3:** Leaf pH values for the three leaf types.

Leaf type	pH
Blue *S*. *uncinata* leaves	4.63 ± 0.03B
Red *S*. *uncinata* leaves	4.55 ± 0.01A
*S*. *kraussiana* leaves	4.52 ± 0.01A

Note: pH values are means ± standard deviation (*n* = 3); A and B show the different significant differences at *P*=0.05 level in SNK test.

**Table 4:** Metal ion contents of the three leaf types.

Sample name	Metal ion content(mg/kg)							
	Cd	Mg	Ca	Mn	Fe	Cu	Zn	Al
Blue S. uncinata leaves	0.04 ± 0.01B	4311.71 ± 340.96B	598.88 ± 41.69A	115.12 ± 8.63A	421.11 ± 22.45B	8.62 ± 0.63B	55.04 ± 4.30A	592.45 ± 14.47B
Red S. uncinata leaves	0.03 ± 0.00A	8134.86 ± 227.00C	919.65 ± 23.63B	139.09 ± 3.70B	308.02 ± 8.97A	5.61 ± 1.23A	58.00 ± 3.26A	316.21 ± 8.44A
S. kraussiana leaves	0.04 ± 0.00AB	3464.87 ± 77.35A	1152.27 ± 19.28C	386.18 ± 10.13C	583.86 ± 7.83C	6.20 ± 0.61A	117.93 ± 1.69B	806.34 ± 4.39C

Note: metal ion content = mean value ± standard deviation (*n* = 3); A, B, and C show the different significant differences at *P*=0.05 level in SNK test.

**Table 5:** Flavonoids in the three leaf types.

Leaf types	Peaks No.	*T*_*R*_ (min)	ESIMS (m/z)	Molecular weight	Molecular formula	Tentative identification	Peak area	The relative content
B	1	9.87	473, 443, 353	563.1369	C_26_H_28_O_14_	6-C-arabinosyl-8-C-	68824.44	0.39
R	2	9.89		563.1397		7-glucosylapigenin	316976.01	2.02
G								
B	2	11.03	473, 443, 353	533.1287	C_25_H_26_O_13_	Apigenin 6,8-di-C-*α*-L-arabinopyranoside	288726.71	1.63
R	5	11.04		533.1292			1666593.14	10.64
G	1	11.03		533.1288			108417.91	1.26
B	3	13.07	287	431.0959	C_21_H_20_O_10_	Genistin	48655.93	0.27
R	6	13.04		431.0971			207658.77	1.33
G								
B	4	18.71	117, 151	285.0407	C_15_H_10_O_5_	Genistein	105164.60	0.59
R								
G								
B	5	21.10	331, 375, 417, 443	537.0793	C_30_H_18_O_10_	Amentoflavone	439318.23	2.48
R	7	21.07		537.0808			1547602.40	9.88
G	2	21.08		537.0817			1374459.97	15.92
B	6	21.18	307, 375	539.0951	C_30_H_20_O_10_	2”,3”-dihydroamentoflavone	529271.52	2.99
R	8	21.15		539.0969			47536.70	0.30
G								
B	7	21.97	331, 375, 417, 443	537.0805	C_30_H_18_O_10_	Robustaflavone	596373.36	3.37
R	10	21.94		537.0817		Tetrahydroamentoflavone	702769.45	4.49
G	4	21.95		537.0816			640841.64	7.42
B	8	22.13	311, 455	541.1114	C_30_H_22_O_10_	2,3,2”,3”-	1160921.65	6.55
R	11	22.09		541.1119			455568.28	2.91
G								
B	9	22.39	307, 375	539.0960	C_30_H_20_O_10_	2,3-Dihydrorobustaflavone	767712.86	4.33
R	12	22.35		539.0970			462224.52	2.95
G	5	22.35		539.0970			43695.79	0.51
B	10	22.61	307, 375	539.0966	C_30_H_20_O_10_	2,3-Dihydroamentoflavone	330804.83	1.87
R	13	22.58		539.0967			305323.38	1.95
G								
B	11	22.88	311, 455	541.1117	C_30_H_22_O_10_	2,3,2”,3”-Tetrahydro robustaflavone	683116.30	3.86
R	14	22.83		541.1129			183554.59	1.95
G								
B	12	23.39	389, 431, 457	551.0960	C_31_H_20_O_10_	Bilobetin	135656.04	0.77
R	15	23.39		551.0977			637558.86	4.07
G	6	23.33		551.0968			892667.03	10.34
B	13	24.16	511, 435, 403	555.1273	C_31_H_24_O_10_	7”-O-methyl-2,3,2”,3”-tetrahydrohinokiflavone	604123.98	3.41
R	16	24.08		555.1298			82994.89	0.53
G								
B	14	24.38	389, 431	551.0971	C_31_H_20_O_10_	Robustaflavone 4′-methyl ether	790017.41	4.46
R	18	24.36		551.0988			974541.47	6.22
G	8	24.36		551.0971			128115.65	1.48
B	15	27.29	533, 519	565.1118	C_32_H_22_O_10_	4′,7”-di-O-methylamentoflavone	754645.71	4.26
R	20	27.26		565.1138			56949.14	0.36
G	9	27.29		565.1130			83280.33	0.96
R	1	8.50	473, 383, 353	593.1502	C_26_H_28_O_14_	6,8-C-diglucosylapigenin	52957.81	0.34
R	3	10.15	473, 443, 353	533.1294	C_25_H_26_O_13_	Apigenin 6,8-di-C-*α*-L-arabinopyranoside	164986.79	1.05
R	4	10.60	473, 443, 353	533.1292	C_25_H_26_O_13_	Apigenin 6,8-di-C-*α*-L-arabinopyranoside	198479.06	1.27
R	9	21.54	405, 473	567.0924	C_31_H_20_O_11_	3‴-O-methylamentoflavone	282241.09	1.80
R	17	24.16	509	553.1126	C_31_H_22_O_10_	Dihydrobilobetin	912746.55	5.83
R	19	24.84	401, 433	553.1143	C_31_H_20_O_10_	Dihydrorobustaflavone 4'-Methyl ether	691000.50	4.41
G	3	21.56	405, 473	539.0963	C_31_H_20_O_11_	3‴-O-methylamentoflavone	20205.96	0.23
G	7	24.18	389, 431	551.0962	C_31_H_20_O_10_	Robustaflavone 4'-methyl ether	465924.15	5.40

Note: B: blue *Selaginella uncinata* leaf; R: red *Selaginella uncinata* leaf; G: *Selaginella kraussiana*; the relative content refers to the proportion of the compound that it occupies in all of the peak materials of the sample.

## Data Availability

The raw data supporting the conclusions of this article will be made available by the authors, without undue reservation.
